The article "Indoor Air Pollution and Blood Pressure in Adult Women Living in Rural China" was published in 2011. Journal: Environ Health Perspect.

# Indoor Air Pollution and Blood Pressure in Adult Women Living in Rural China

**DOI:** 10.1289/ehp.1003371

**Published:** 2011-07-01

**Authors:** Jill Baumgartner, James J. Schauer, Majid Ezzati, Lin Lu, Chun Cheng, Jonathan A. Patz, Leonelo E. Bautista

**Affiliations:** 1 Institute on the Environment, University of Minnesota, St. Paul, Minnesota, USA; 2 Department of Population Health Sciences,; 3 Nelson Institute for Environmental Studies, and; 4 Environmental Chemistry and Technology Program, University of Wisconsin, Madison, Wisconsin, USA; 5 MRC-HPA Centre for Environment & Health, Department of Epidemiology and Biostatistics, School of Public Health, Imperial College London, London, United Kingdom; 6 Yunnan Provincial Centers for Disease Control and Prevention, Kunming, Yunnan, People’s Republic of China; 7 Institute for Global Health, University of Wisconsin, Madison, Wisconsin, USA

**Keywords:** biomass, blood pressure, cardiovascular health, China, household air pollution, indoor air pollution, particulate matter, solid fuels

## Abstract

Background: Almost half of the world’s population uses coal and biomass fuels for domestic energy. Limited evidence suggests that exposure to air pollutants from indoor biomass combustion may be associated with elevated blood pressure (BP).

Objective: Our aim was to assess the relationship between air pollution exposure from indoor biomass combustion and BP in women in rural China.

Methods: We measured 24-hr personal integrated gravimetric exposure to fine particles < 2.5 µm in aerodynamic diameter (PM_2.5_) and systolic BP (SBP) and diastolic BP (DBP) in the winter and summer among 280 women ≥ 25 years of age living in rural households using biomass fuels in Yunnan, China. We investigated the association between PM_2.5_ exposure and SBP and DBP using mixed-effects models with random intercepts to account for correlation among repeated measures.

Results: Personal average 24-hr exposure to PM_2.5_ ranged from 22 to 634 µg/m^3^ in winter and from 9 to 492 µg/m^3^ in summer. A 1-log-µg/m^3^ increase in PM_2.5_ exposure was associated with 2.2 mm Hg higher SBP [95% confidence interval (CI), 0.8 to 3.7; *p* = 0.003] and 0.5 mm Hg higher DBP (95% CI, –0.4 to 1.3; *p* = 0.31) among all women; estimated effects varied by age group. Among women > 50 years of age, a 1-log-µg/m^3^ increase in PM_2.5_ exposure was associated with 4.1 mm Hg higher SBP (95% CI, 1.5 to 6.6; *p* = 0.002) and 1.8 mm Hg higher DBP (95% CI, 0.4 to 3.2; *p* = 0.01). PM_2.5_ exposure was positively associated with SBP among younger women, but the association was not statistically significant.

Conclusion: PM_2.5_ exposure from biomass combustion may be a risk factor for elevated BP and hence for cardiovascular events. Our findings should be corroborated in longitudinal studies.

The article "Indoor Air Pollution and Blood Pressure in Adult Women Living in Rural China" was published in 2011. Journal: Environ Health Perspect.

Biomass (wood, crop residues, and animal dung) and coal are the primary fuels for almost half the world’s population, who live mostly in low-income regions (Smith et al. 2004). These fuels are often burned inside poorly ventilated spaces with thermally inefficient stoves (Bruce et al. 2000; Smith 1987) that emit a complex pollutant mixture of particulate matter (PM) and other toxic compounds at concentrations much higher than most urban ambient pollution levels (Smith et al. 2004). The effects of indoor air pollution on chronic obstructive pulmonary disease and lung cancer (coal use only) in adults and pneumonia in children are well documented (Bautista et al. 2009; Dherani et al. 2008; International Agency for Research on Cancer 2010; Kurmi et al. 2010; Padmavati and Pathak 1959; Smith et al. 2004). Limited evidence also suggests an association with tuberculosis (Lin et al. 2007), cataracts (Mohan et al. 1989; Zodpey and Ughade 1999), and low birth weight (Boy et al. 2002).

Exposures to ambient air pollution and tobacco smoke have been associated with increased risk of myocardial infarction, stroke, and cardiovascular mortality (Barnoya and Glantz 2005; Brook et al. 2010; U.S. Department of Health and Human Services 2006). Several mechanisms have been proposed for these cardiovascular effects, including PM-induced increases in blood pressure (BP) (Pope et al. 2004). Human experiments (Brook et al. 2009; Langrish et al. 2009; Urch et al. 2005) and observational studies (Auchincloss et al. 2008; Brook et al. 2011; Choi et al. 2007; Delfino et al. 2010; Dvonch et al. 2009; Ibald-Mulli et al. 2001; Kannan et al. 2010; Linn et al. 1999; Liu et al. 2009; Zanobetti et al. 2004) suggest that ambient air pollution exposure could raise systolic BP (SBP) and diastolic BP (DBP), although other studies failed to replicate these findings (Brauer et al. 2001; Ebelt et al. 2005; Harrabi et al. 2006; Ibald-Mulli et al. 2004; Jansen et al. 2005; Madsen and Nafstad 2006).

Although ambient PM studies combined with toxicological studies of woodsmoke exposure (Naeher et al. 2007) suggest a potential role of indoor air pollution in BP elevation, there are limited epidemiologic data in support of this hypothesis. Only a randomized intervention study in Guatemalan women demonstrated that transitioning from an open fire to an improved biomass stove was associated with lower BP (McCracken et al. 2007). The lack of epidemiologic data on the cardiovascular health effects of indoor air pollution limits our ability to assess its full public health impact (Smith and Peel 2010). For example, the most recent World Health Organization (WHO) Comparative Risk Assessment did not attribute cardiovascular outcomes to household use of solid fuels (WHO 2009).

The article "Indoor Air Pollution and Blood Pressure in Adult Women Living in Rural China" was published in 2011. Journal: Environ Health Perspect.

In the present study we assessed the relationship between personal exposure to PM from biomass combustion and BP in women in rural China. Our study is particularly relevant to China, which has low incidence of ischemic stroke but high incidence of hemorrhagic stroke relative to other regions (Zhang et al. 2003).

## Materials and Methods

*Study location and population.* The study took place in six villages in northwestern Yunnan province, China (N 26°52´, E 100°06´). Most participants are members of the Naxi minority group and have similar socioeconomic backgrounds and dietary habits. All households used biomass for cooking or heating. Ninety-four percent of households used biomass as their primary cooking fuel, but all also used at least one “improved” fuel (liquefied petroleum gas, biogas, or electricity). Space heating with wood logs or wood charcoal is common during winter (98% of households).

*Participant recruitment.* We recruited 280 women from 235 rural households. Women who were current or former cigarette smokers or pregnant at the time of the study were excluded. Local field staff explained the objectives and methods of the study to village women’s groups and identified eligible participants with assistance from village leaders. Women interested in participation were read a consent form by field staff, and all provided oral informed consent. The study was approved by the Health Sciences Institutional Review Board at the University of Wisconsin-Madison and the Yunnan Provincial Health Bureau, Kunming, China. Data collection took place in winter (December 2008–February 2009) and summer (June–August 2009).

*Personal PM_2.5_ exposure measurement.* We measured 24-hr personal integrated gravimetric exposure to fine particles < 2.5 μm in aerodynamic diameter (PM_2.5_) in winter and summer. PM_2.5_ is widely considered the best indicator of adverse health effects from combustion-related pollution (Pope and Dockery 2006). Sampling occurred every day of the week, except holidays when cooking periods are unusually long and hence an inappropriate measure of usual exposure. In each season, approximately 10% of participants were randomly selected for 24-hr measurements of PM_2.5_ exposure on 2 consecutive days to assess day-to-day exposure variation.

Participants wore a portable, battery-operated pump (Apex Pro; Casella CEL, Bedford, UK) in a small waistpack (< 1 kg) for gravimetric PM_2.5_ measurements. Field staff instructed participants to perform routine daily activities and wear the waistpack at all times. However, they could place the waistpack within 1 m while resting or sleeping and within 2 m during activities when wearing it was very inconvenient or impossible (i.e., bathing). To monitor compliance, field staff conducted daily visits to participants’ homes and attached pedometers to the waistpacks.

The article "Indoor Air Pollution and Blood Pressure in Adult Women Living in Rural China" was published in 2011. Journal: Environ Health Perspect.

The pump was connected to a Slaton aluminum cassette (BGI Inc., Waltham, MA, USA) loaded with a 37-mm Teflon filter (2.0-μm pore size; SKC Inc., Eighty Four, PA, USA) and attached downstream from a GK2.05 (KTL) cyclone with a 2.5-µm aerodynamic-diameter cut point (BGI Inc.) when operated at 4 L/min ± 10%. The air-flow rate through the filters was measured at the beginning and end of each sampling period using a calibrated rotameter. Because of the high altitude of the study site, we corrected for atmospheric pressure changes during rotameter calibration in Madison, Wisconsin (Caplan 1985).

The Teflon filters were weighed pre- and postsampling at the Wisconsin State Hygiene Laboratory after being conditioned in a temperature- and humidity-controlled environment (23°C and 40%) for at least 24 hr and were statically discharged using a polonium source. We weighed each filter in triplicate using a microbalance (MX-5; Mettler Toledo, Columbus, OH, USA) with a readability of 1 μg. If the initial three weights differed by > 5 μg (2% of filters), we reweighed the filter until a stable weight was achieved. The average of the three closest weights was used as the final weight for analysis. The zero and span of the balance were checked after every batch of 20 samples.

For quality control and to assess potential contamination, 10% field blank filters were placed in identical cassettes, subject to the same field conditions, and analyzed using the same protocol as the sample filters. We performed blank correction by subtracting the median mass of field blanks collected seasonally in each village and obtained the mass concentration by dividing the blank-corrected-mass by the corresponding Teflon filter sample volume. The mean mass of blanks was 0.72 µg [95% confidence interval (CI), –2.3 to 3.78]. All pump flow rates were ± 8% of the target and 90% of samples ran within 2 hr of the target 24-hr sampling period. Of the 652 PM samples collected, we excluded five from the analysis because of equipment failure or filter damage.

*BP measurements.* We conducted home BP measurements immediately before and after each participant’s PM_2.5_ personal exposure monitoring period using an automated device (Omron-705CP; Omron Corp, Tokyo, Japan), that has been validated against a mercury sphygmomanometer according to the revised protocol of the British Hypertension Society (O’Brien et al. 1996). The mean and median times between PM monitoring completion and BP measurement were 15 min and 6 min, respectively. After ≥ 5 min of quiet rest, three consecutive BP measures were taken 1 min apart on the supported right arm of the seated participant in accordance with standard recommendations (Pickering et al. 2005). We also recorded the date, time, and ambient air temperature and whether the participant had consumed caffeine in the previous hour. The average of the last two BP measures was used as the subject’s final BP estimate. Women with average SBP ≥ 140 mm Hg and/or DBP ≥ 90 mm Hg or using antihypertensive medication were considered hypertensive.

The article "Indoor Air Pollution and Blood Pressure in Adult Women Living in Rural China" was published in 2011. Journal: Environ Health Perspect.

*Questionnaires and other measurements.* We collected sociodemographic and health information for each participant: age, education, current medication use, and cardiovascular history, including physician-diagnosed diabetes, kidney disease, myocardial infarction, stroke, or hypertension. We asked participants if they had experienced difficulty in carrying out daily activities or work because of illness in the past 3 months and to describe their health compared with women of similar age (categorized as excellent, good, fair, or poor). Passive smoking status was obtained by asking about the number of active smokers in the participant’s household and the average number of cigarettes smoked per day by each smoker. We assigned a composite socioeconomic status (SES) score to each household, which was constructed from data on the ownership of 17 household assets using principal components analysis (Filmer and Pritchett 2001). In developing countries, asset-based measures of SES are considered more robust and less-biased indicators of long-term economic status than self-reported income or consumption of goods (Sahn and Stifel 2003).

For each participant, we measured height (centimeters), weight (kilograms), and waist circumference (centimeters) and calculated body mass index (BMI) by dividing weight (kilograms) by height (meters squared). Physical activity was assessed by using both 24-hr pedometer measurement and estimation of the time per week engaged in different activity levels using the WHO Global Physical Activity Questionnaire (WHO 2006). Using these activities, we calculated a weekly metabolic equivalent task score for each participant. The validity of this questionnaire in assessing physical activity in rural populations in developing countries is described elsewhere (Bull et al. 2009). Finally, we estimated individual 24-hr salt intake by weighing the salt container of each household before and after a 24-hr period, taking the difference between the two measures, and dividing it by the number of residents in the household.

The article "Indoor Air Pollution and Blood Pressure in Adult Women Living in Rural China" was published in 2011. Journal: Environ Health Perspect.

*Analysis of PM–BP association.* We log-transformed PM_2.5_ concentrations to improve normality and variance homogeneity, supported by evidence suggesting a log-linear exposure–response relationship between PM and cardiovascular outcomes (Pope et al. 2009). In the first analysis, we used mixed-effects models with random intercepts at the individual, household, and village level to assess the independent effect of PM_2.5_ exposure on BP and adjust for time-invariant factors in the same individual, within participants in the same household, and within the same village (Laird and Ware 1982). Individual-level random effect estimates accounted for measurements in two seasons. Within each season, we used the first observation for individuals with repeated measurements, because only a subset of participants had repeated within-season measurements. We analyzed the effect of PM_2.5_ exposure on both postexposure BP and average pre- and postexposure BP in separate regression models.

We estimated the following regression equation:

γ*_ifkj_* = µ + β^ˆ^_1_ln(PM_2.5_)*_ifkj_* + γ*x_ifkj_*   + η*z_ifk_* + α*_ifk_* + *h_fk_* + ν*_k_* + ε*_ij_*, [1]

where *y* denotes either SBP or DBP in individual *i*, in household *f,* in village *k,* in season *j*; *μ* represents a constant; β^ˆ^_1_1n(*PM*_2.5_) is the effect size estimate per ln(PM_2.5_) exposure; γ*x_ifkj_* represents the time-varying covariates (i.e., day and time of BP measurement, ambient air temperature, physical activity, caffeine intake, and self-reported health); η*z_ifk_* denotes covariates that are time-invariant or that changed only minimally during the study period (i.e., age, years of education, waist circumference, SES, salt intake, passive smoking); α*_ifk_* represents the random intercept with the distribution ~ *n*(0,σ_a_^2^); *h_fk_* represents the random effects at the household level with the distribution ~ *n*(0,σ_h_^2^); ν*_k_* represents the random effects at the village level with the distribution ~ *n*(0,σ_v_^2^); and ε*_ij_* is the error term with the distribution ~ *n*(0,σ^2^).

We retained variables in the final model if they were associated with BP at *p* < 0.10 or if they changed the effect of PM exposure on BP by ≥ 10%. We also assessed effect size modification by age, BMI dichotomized as obese or overweight (BMI ≥ 25 kg/m^2^) versus normal weight or underweight (BMI < 25 kg/m^2^), hypertension status, and passive smoking by including the interaction between personal PM exposure and the potential effect modifier in the mixed-effects models. If the interaction was statistically significant (*p* < 0.05), we conducted separate analyses corresponding with each group.

The article "Indoor Air Pollution and Blood Pressure in Adult Women Living in Rural China" was published in 2011. Journal: Environ Health Perspect.

Finally, we used our estimated mixed-effects log-linear regression models to predict the average SBP and DBP in the population (i.e., marginal means). For this purpose, all covariates in the models were kept at their average value except for PM_2.5_ exposure, which was allowed to vary within the exposure range that we observed in our study population (StataCorp 2009).

In a second analysis, we took advantage of the within-season repeated PM_2.5_ measurements in about 10% of participants to account for the day-to-day variability in exposure. For this purpose, we used a covariate measurement error (CME) model (Rabe-Hesketh et al. 2003). The CME model predicts an individual’s corrected usual exposure from a mixed-effects model and then uses the corrected exposure value in a multivariate regression model. Participants with only one PM_2.5_ value still contribute to the analysis, under the assumption that the sample with repeated exposure measurements was drawn at random (i.e., that repeated measures of PM_2.5_ are missing at random). For the CME analysis, we used a “wrapper” command that uses the adaptive quadrature method implemented through the “gllamm” command (Rabe-Hesketh et al. 2002).

All statistical analyses were performed in STATA 11 (StataCorp, College Station, TX, USA).

## Results

We enrolled 280 women 25–90 years of age (mean age, 51.9 years). Of these, 196 participated in both the winter and summer, 66 only in the winter, and 18 only in the summer. Most declines to participate in both evaluations were due to the farming season schedule. Most participants had some form of formal education (52% primary and 31% secondary school). The mean (± SD) BMI and waist circumference among participants were 23 ± 4 kg/m^2^ and 82 ± 9 cm, respectively. Seventeen percent were overweight (BMI, 25–29.9 kg/m^2^), and 4% were obese (BMI ≥ 30 kg/m^2^).

Personal 24-hr exposure to PM_2.5_ ranged from 9 to 492 µg/m^3^ [interquartile range (IQR), 61 µg/m^3^; median, 52 µg/m^3^] in summer and 22 to 634 µg/m^3^ (IQR, 120 µg/m^3^; median, 105 µg/m^3^) in winter. The 24-hr geometric mean PM_2.5_ exposure in summer was 55 µg/m^3^ (95% CI, 49 to 62) and increased to 117 µg/m^3^ (95% CI, 107 to 128) in winter.

None of the participants reported kidney disease, a previous myocardial infarction, or stroke, and < 1% (*n* = 2) had physician-diagnosed diabetes. Mean SBP and DBP were 120 (95% CI, 118 to 122) and 72 mm Hg (95% CI, 71 to 73), respectively. Thirteen percent (*n* = 37) of participants were hypertensive; 78% (*n* = 29) of hypertensive women were unaware of their status, and only 17% (*n* = 6) were taking antihypertensive medication. Among women with measurements in both seasons, SBP was significantly higher in winter than in summer (120 mm Hg; 95% CI, 117 to 122 vs. 116 mm Hg; 95% CI, 113 to 118; *p* < 0.001), with no seasonal difference in DBP (73 mm Hg; 95% CI, 71 to 74 vs. 73 mm Hg; 95% CI, 71 to 74; *p* = 90). Similar to observations in other populations (Lawes et al. 2004), SBP increased with age, whereas DBP increased until approximately 60 years of age and then slightly decreased thereafter.

The article "Indoor Air Pollution and Blood Pressure in Adult Women Living in Rural China" was published in 2011. Journal: Environ Health Perspect.

*PM–BP associations.* Personal PM_2.5_ exposure was positively associated with postexposure measurement of SBP and DBP (Table 1). A 1-log-µg/m^3^ increase in PM_2.5_ exposure was associated with 2.2 mm Hg higher SBP (95% CI, 0.8 to 3.7; *p* = 0.003) and 0.5 mm Hg higher DBP (95% CI, –0.4 to 1.3; *p* = 0.31) among all women; however, the estimated effect was dependent on age. We observed evidence of an age-by-exposure interaction using 10-year age groups but lacked sufficient statistical power to estimate effects with reasonable precision. We therefore dichotomized age as 25–50 years and > 50 years based on biological parameters and the relative increase in cardiovascular risk beginning in the fifth decade of life (Mackay and Mensa 2004). The PM–BP associations were not significantly modified by BMI, hypertension status, or passive smoking.

**Table 1:** Crude and multivariate adjusted effects of personal PM_2.5_ exposure on BP by age.

Crude effects*a*			Adjusted effects*b*		
Age (years)	*n*	Difference (mm Hg) (95% CI)	*p*-Value	Difference (mm Hg) (95% CI)	*p*-Value
SBP										
25–50		142		1.6 (0.4 to 2.8)		0.008		0.7 (–0.8 to 2.1)		0.35
> 50		138		4.1 (1.7 to 6.5)		0.001		4.1 (1.5 to 6.6)		0.002
All		280		2.7 (1.4 to 4.1)		< 0.001		2.2 (0.8 to 3.7)		0.003
DBP										
25–50		142		0.1 (–1.1 to 1.3)		0.88		–0.6 (–1.7 to 0.5)		0.25
> 50		138		1.2 (–0.1 to 2.4)		0.06		1.8 (0.4 to 3.2)		0.01
All		280		0.0 (–0.8 to 0.8)		0.98		0.5 (–0.4 to 1.3)		0.31
The effect is the estimated difference in BP associated with a 1-unit increase in the log of PM_2.5_. **a**Results are from univariate mixed-effects models. **b**Adjusted for age, waist circumference, physical activity, SES, salt intake, day of the week, time of day, and average ambient temperature, with all variables modeled as continuous except day of the week; results are from multivariate mixed-effects models.										

In the crude analysis, a 1-log-µg/m^3^ increase in PM_2.5_ exposure was associated with 2.7 mm Hg higher SBP; (95% CI, 1.4 to 4.1; *p* < 0.001); the effect was larger in women > 50 years of age (4.1 mm Hg; 95% CI, 1.7 to 6.5; *p* = 0.001) than in women 25–50 years of age (1.6 mm Hg; 95% CI, 0.4 to 2.8; *p* = 0.008) (Table 1). This pattern of a stronger association in older women persisted after adjusting for other risk factors, but after adjustment the association was no longer significant in younger women (0.7 mm Hg; *p* = 0.35). The interaction between PM_2.5_ and age group on SBP was statistically significant (*p* = 0.03).

The article "Indoor Air Pollution and Blood Pressure in Adult Women Living in Rural China" was published in 2011. Journal: Environ Health Perspect.

We observed similar results for DBP, with both crude and adjusted estimates indicating a nonsignificant effect of PM_2.5_ among young women and significantly higher DBP among older women (Table 1). After adjusting for other variables, a 1-log-µg/m^3^ increase in PM_2.5_ exposure was associated with 1.8 mm Hg higher DBP in women > 50 years of age (*p* = 0.01). The interaction between PM_2.5_ and age group was also significant for DBP (*p* = 0.01).

An average woman > 50 years of age exposed to the average PM_2.5_ level in our study population (~ 100 µg/m^3^) had an estimated SBP and DBP of 128 and 76 mm Hg, respectively (Figure 1). However, if the same woman was exposed to PM_2.5_ concentrations in the upper decile of our exposure distribution (~ 500 µg/m^3^), her estimated SBP and DBP increased to 135 and 79 mm Hg, respectively.

**Figure 1:** Average SBP and DBP in the population by level of personal exposure to PM_2.5_ and age.**∆ indicates the difference in blood pressure by a 1-unit increase in the log of PM_2.5_ (as shown in Table 1). Average SBP and DBP in the population (marginal means) were predicted from mixed-effects log-linear regression models (Table 1) using the mean values of age, waist circumference, pedometer steps, SES, salt intake, time of day, and ambient air temperature for the population and the range of PM_2.5_ exposure observed in our study population. Mean ages were 40 years for the 25–50 age group and 64 years for the > 50 age group. The mean values for waist circumference, pedometer steps, and salt intake for all women were 82 cm, 7,600 steps, and 6 g, respectively, and did not differ between age groups.

Our findings did not change when we used average BP (i.e., the mean of the before and after exposure measurements of BP) as the dependent variable or when we excluded women with diabetes (*n* = 2) or those who were potentially noncompliant (waistpack pedometer < 500; *n* = 12) from the analysis (results not reported).

Using the CEM model to account for day-to-day variability in PM_2.5_ exposure, the estimated effect of a 1-log-µg/m^3^ increase in PM_2.5_ exposure on SBP decreased from 4.1 to 2.1 mm Hg in women > 50 years of age but remained statistically significant (95% CI, 1.9 to 2.9; *p* < 0.001; Table 2). In contrast, the effect estimate for DBP in older women remained roughly the same (2.3 mm Hg; 95% CI, 0.0 to 4.7; *p* = 0.05). The effect estimates for SBP and DBP increased considerably among younger women but remained nonsignificant.

The article "Indoor Air Pollution and Blood Pressure in Adult Women Living in Rural China" was published in 2011. Journal: Environ Health Perspect.

**Table 2:** Estimated effects of personal pollution exposure (PM_2.5_, µg/m^3^) on BP adjusted for CME.

Age (years)	∆SBP (mm Hg) (95% CI)	*p*-Value	∆DBP (mm Hg) (95% CI)	*p*-Value
25–50 (*n* = 142)		4.4 (–6.4 to 15.2)		0.43		1.3 (–6.5 to 9.2)		0.74
> 50 (*n* = 138)		2.1 (1.9 to 2.9)		0.001		2.3 (0.0 to 4.7)		0.05
Effect estimates are from a CME model based on multilevel regression and are adjusted for age, waist circumference, physical activity, SES, salt intake, day of the week, time of day, and average ambient temperature, with all variables modeled as continuous except day of the week.								

## Discussion

Using data on both personal exposure to PM_2.5_ and BP measurements in two seasons, we found a significant positive association between increased exposure to PM_2.5_ and both SBP and DBP. A 1-log-µg/m^3^ increase in PM_2.5_ exposure was associated with 4.1 mm Hg higher SBP (95% CI, 1.5 to 6.6) and 1.8 mm Hg higher DBP (95% CI, 0.4 to 3.2) in women > 50 years of age. PM_2.5_ exposure was positively associated with SBP among younger women, but the association was not statistically significant. Our results are consistent with a previous epidemiologic study on indoor biomass smoke and BP (McCracken et al. 2007), which found that use of improved cooking stoves, resulting in lower PM exposure, was associated with 3.7 mm Hg lower SBP (*p* = 0.10) and 3.0 mm Hg lower DBP (*p* = 0.02) relative to a traditional open-fire control group. Further, in our study we had personal PM exposure data and could thus estimate the exposure–response relationship.

Several studies on ambient air pollution have also shown an association between PM_2.5_ and BP. However, in those studies PM_2.5_ likely originated from sources other than biomass combustion, and the PM exposure levels were considerably lower than in our study. Among the few studies with personal PM_2.5_ exposure measurement, Liu et al. (2009) found a 3.7-mm Hg (95% CI, 0.6 to 6.7) increase in SBP per 7.1-µg/m^3^ increase in PM exposure in elderly subjects, and Brook et al. (2010) observed a 1.4-mm Hg (95% CI, 0.8 to 2.1) elevation in SBP per 10-µg/m^3^ increase in PM exposure in a community sample of adults. The SBP effects observed in those studies were roughly comparable to those estimated for older women in our study. Other studies with ambient or household PM exposure measurements found that PM_2.5_ was positively associated with higher BP across 1- to 2-day time lags (Dvonch et al. 2009; Kannan et al. 2010; Lin et al. 2009), but the PM effect was stronger than the one observed in our study.

The article "Indoor Air Pollution and Blood Pressure in Adult Women Living in Rural China" was published in 2011. Journal: Environ Health Perspect.

The notable strengths of our study include measurment of personal exposure, data on exposure and BP collected in summer and winter, and adjustment for important risk factors for increased BP including age, obesity, physical activity, and salt intake. Although our method of estimating salt intake has not been validated previously and was measured at the household level, it was selected based on the local logistical and cultural context. Specifically, measurement of urinary sodium was logistically impossible, and we are not aware of a previously validated food frequency questionnaire for a rural Naxi population. Residual confounding for salt intake or other covariates may remain. However, it is unlikely that these or other unmeasured covariates are strong confounders in our mixed-effects models, given the relative homogenous distribution of risk factors for elevated BP in our study population, which facilitates control of unmeasurable or difficult-to-measure risk factors.

We used 24-hr PM_2.5_ exposure measurement because data on longer-term seasonal exposure were not feasible given resource and time constraints. However, our overall conclusions about the PM–BP relationship were robust after accounting for day-to-day variation in PM_2.5_ exposure based on repeated 24-hr exposure measurements. Field staff did not observe any instances where wearing the waistpack impeded the normal physical activity of the participant; however, we cannot completely eliminate the possibility. Technologies that can more easily measure long-term PM exposure would greatly benefit epidemiologic research on indoor air pollution and health.

An important limitation of this study is its cross-sectional design. Cooking with biomass is a long-term behavior; thus, 24-hr PM exposure is a measure that is usual except for day-to-day variability. In addition, an individual’s BP is not likely to affect PM exposure, given that increases in BP are usually asymptomatic. Although some occult cardiac disease may exist in our study population, it is unlikely that asymptomatic conditions would influence exposure to PM. It is possible that poor health status, some of which may be attributable to undiagnosed cardiovascular comorbidities, may lead women to reduce their PM exposure. However, adjusting for self-reported health status in the regression models did not alter our findings. Similarly, unreported use of medications such as oral contraceptives or antidepressants cannot explain our findings, because their use is extremely rare in this population (Hardee et al. 2004; Parker et al. 2001).

In our mixed-effects models, 24-hr pedometer measurement was the only marker of physical activity associated with BP. Travel between households, agricultural fields, and the local market often involves walking alongside the major highway running through the study site and may increase exposure to traffic emissions. Therefore, number of pedometer steps may be a marker of physical activity and/or exposure to traffic pollution in our study. Similarly, our use of personal PM_2.5_ mass prevents us from studying the relative contribution of different PM constituents or sources on the observed BP effects.

The article "Indoor Air Pollution and Blood Pressure in Adult Women Living in Rural China" was published in 2011. Journal: Environ Health Perspect.

In addition, although our use of 24-hr average personal PM exposure provides a more useful exposure profile than household or proxy measurements (i.e., cooking frequency or primary fuel type) for epidemiologic analysis, it does not account for high-intensity pollution exposure periods that may occur, for instance, while cooking or starting a fire. As previously hypothesized (Ezzati et al. 2000), this may systematically underestimate exposure for some women. However, if high- intensity exposure positively modifies the effect of PM exposure on BP, our findings would underestimate the health effects in the overall population using biomass fuels.

Previous studies indicate that transitioning from an open fire to an improved (i.e., enclosed and vented) wood cookstove (Albalak et al. 2001), liquefied petroleum gas (Naeher et al. 2000), or wood charcoal (Ezzati and Kammen 2002) can result in at least a 1-log-µg/m^3^ reduction in indoor PM. Based on our results, such a change could result in approximately 4 mm Hg lower SBP among older women. Strong evidence suggests that risk of cardiovascular mortality increases progressively and linearly with increasing BP at levels as low as 115 mm Hg SBP and 75 mm Hg DBP in Western and Asian populations (Lawes et al. 2004; Lewington et al. 2002). Based on results from Lawes et al. (2003), we estimate that 4 mm Hg lower SBP on a population level would result in an 18% (95% CI, 15 to 21) decrease in coronary heart disease and a 22% (95% CI, 21 to 24) decrease in stroke among Asian women 50–59 years of age. Considering that biomass fuels are the primary domestic energy source for > 2 billion people globally (Smith et al. 2004), the potential cardiovascular benefit of transitioning to cleaner-burning stoves and fuels on a macro level would be considerable. For example, based on the published mortality data for Chinese women, an 18% decrease in coronary heart disease and 22% decrease in stroke would account for up to 230,900 fewer deaths per year in Chinese women > 50 years of age.

The log-linear association in our study has important implications for the relative benefits of PM exposure reductions at different points along the exposure–response curve (Smith and Peel 2010), notably that the same absolute reduction at lower exposure levels may have greater population health benefit. For instance, based on our results, the cardiovascular benefit of transitioning from an improved biomass cookstove to liquefied petroleum gas may be greater than switching from an open fire to an improved biomass cookstove, even if the absolute emissions reduction in these two intervention scenarios is identical. Obviously, there are also considerable differences in cost and feasibility in these two scenarios that require consideration. Intervention options would benefit from cost–benefit analyses of different improved stove and fuel scenarios that incorporate these factors.

The article "Indoor Air Pollution and Blood Pressure in Adult Women Living in Rural China" was published in 2011. Journal: Environ Health Perspect.

We cannot determine the duration of PM effects on BP or whether reductions in PM lead to decreases in BP, as has been shown for salt in randomized trials (He and MacGregor 2002). Previous studies have shown that PM-triggered elevations in BP may occur acutely (2 hr) (Urch et al. 2005) in a more delayed fashion (1–5 days) (Zanobetti et al. 2004) and in the long term (McCracken et al. 2007). A change in autonomic tone is the most likely mechanism for short-term increases in BP minutes after PM inhalation (Brook et al. 2009). PM inhalation favors withdrawal of vagal activity and stimulation of the sympathetic nervous system (Narkiewicz et al. 1998), resulting in systemic vasoconstriction, increased cardiac output, and acute change in BP (Brook 2005).

The stronger estimated effect among older women in our study may be attributable to long-term oxidative stress and systemic inflammation due to lifetime PM exposure. PM inhalation has been shown to cause oxidative stress (Barregard et al. 2006) as well as systemic inflammation (Pope and Dockery 2006), which is associated with the development of hypertension (Bautista et al. 2005). Long-term BP effects of PM exposure could also be the result of a resetting of BP-regulating mechanisms to higher levels as a consequence of repeated acute increases in BP after PM inhalation. Although underlying cardiovascular disease has been proposed as a potential driver of an age-by-exposure interaction (Brook et al. 2010), it does not likely explain our results given the low cardiovascular disease prevalence in our study population. A recent study found the opposite, with stronger estimated effects of PM on BP in women < 50 years of age (Dvonch et al. 2009), but this may be attributable to use of BP medication in older women, resulting in a dampening of the effect of PM on BP in this age group.

## Conclusion

Our study shows that personal PM_2.5_ exposure is positively associated with both SBP and DBP among adult women, particularly in those > 50 years of age. Although our findings should be confirmed in prospective cohort studies, they suggest that cardiovascular diseases may be an important component of the public health burden of indoor cooking and heating with biomass fuels. Issues of energy and indoor air pollution should therefore be considered in the formulation of policies and interventions aimed at reducing the cardiovascular disease burden in China and other countries where domestic use of biomass fuels is common.
